# Natural Adrenocorticotropic Hormone (ACTH) Relieves Acute Inflammation in Gout Patients by Changing the Function of Macrophages

**DOI:** 10.1155/2022/9241835

**Published:** 2022-03-22

**Authors:** Rui Xu, Li Zhao, Jiyu Liu, Lin Cao, Tianyi Zhao, Yiyun Yu, Dandan Xuan, Weiguo Wan, Yu Xue, Hejian Zou

**Affiliations:** ^1^Division of Rheumatology, Huashan Hospital, Fudan University, Shanghai 200040, China; ^2^Human Phenome Institute, Fudan University, Shanghai 201203, China; ^3^Institute of Rheumatology, Immunology and Allergy, Fudan University, Shanghai 200040, China

## Abstract

Gout is a common arthritis caused by deposition of monosodium urate crystals. Macrophage is crucial in the process of monosodium urate (MSU)-induced inflammation. Although it has been reported that adrenocorticotropic hormone (ACTH) in nature can be used to cure urarthritis, the mechanism concerning macrophage is still not clear. However, gout patients manifest other complications, such as hypertension, diabetes, chronic kidney disease, and hormone intolerance, which limit efficacy of some of these first-line drugs. Therefore, this study aims to explore how natural ACTH can alleviate urarthritis through functional changes in macrophage. We analyzed the variations in VAS pain scores of five patients, knowing the time of action and detecting the level of cortisol and ACTH in patients 24 hours after the application of ACTH. The effect of natural ACTH on joint inflammation and the level of cortisol in blood in the mouse model was evaluated by studies in vivo. In vitro studies, we evaluated the effect of natural ACTH on macrophages and revealed different functions of ACTH and dexamethasone on macrophages in the transcriptional level. In patients with acute gout, natural ACTH can quickly alleviate pain and does not affect the level of cortisol and ACTH. Natural ACTH is able to ease the swelling and inflammatory cell infiltration caused by arthritis, without changing the level of cortisol. Besides, natural ACTH in vitro can alleviate acute gouty inflammation by regulating phagocytosis and polarization of macrophage, which also exerts different effects on the transcription of some related genes. Natural ACTH is able to alleviate acute gouty inflammation by regulating macrophage, and this effect differs from that of dexamethasone at the transcriptional level.

## 1. Introduction

Gout, a type of crystal-related arthropathies caused by deposition of monosodium urate (MSU) in joints, is directly associated with hyperuricemia resulting from purine metabolic disorders and/or decreased excretion of uric acid, making it a kind of metabolic rheumatism [1]. Apart from joint damage, patients with gout may also be predisposed to kidney disease and other metabolic syndromes, such as hyperlipidemia, hypertension, diabetes, and coronary heart disease [2]. The American College of Rheumatology Guidelines for the Management of Gout 2020 [3] have strongly recommended colchicine, nonsteroidal anti-inflammatory drugs (NSAIDs), or corticosteroids (oral, intrajoint, or muscle injection) as the first-line drugs for the treatment of acute gout.

ACTH, a type of polypeptide hormone secreted by the pituitary glands of vertebrates, promotes tissue hyperplasia of the adrenal cortex as well as production and secretion of cortical hormone. Notably, natural ACTH, whose production and secretion are directly regulated by corticotropin-releasing factors (CRF) secreted from the hypothalamus [4], is an important hormone that maintains the normal morphology and function of the adrenal gland. At present, natural ACTH is commonly used to treat collagenosis like rheumatoid arthritis [5, 6] and systemic lupus erythematosus [7, 8]. However, it is not a first-line drug for the treatment of acute gout. In fact, ACTH was first used to treat acute gout more than half a century ago [9]. Since then, some studies have showed that ACTH not only generates equal efficacy but also has similar safety profiles to those of NSAIDs and steroids [10–12]. For example, gout patients treated with ACTH-exhibited stable levels of blood pressure and serum potassium [13], without showing apparent adverse reactions. Another study showed that ACTH was efficacious in gout patients who had various complications or who could not bear standard treatment, with efficiencies as high as 77.9–100% [14].Research evidence has shown that natural ACTH can effectively improve kidney function and have a lipid-lowering effect relative to traditional medicines like NSAIDs and corticosteroids [15]. Besides, ACTH has also been used to treat patients with hypoadrenia, glucocorticoid resistance, and even those with contraindications. Currently, natural ACTH is seldom used for the treatment of acute gout, owing to the high cost of formulation in most countries.

Additional research evidence has demonstrated that inflammatory factors like IL-I*β*, secreted during the process of acute gouty arthritis, stimulate the anterior pituitary gland to generate natural ACTH. It subsequently binds to the receptor, MC-2R, on adrenal, thereby inducing secretion of corticosteroid, and finally downregulating corresponding inflammatory factors [14, 15]. Recent research findings have revealed the underlying mechanism of acute gout. For example, ACTH was shown to bind to receptor MC-3R on macrophages to stimulate melanocortin transduction and suppress secretion and release of chemokines, which regulate the accumulation of neutrophils [14], thereby alleviating inflammation. Notably, ACTH exhibited fewer adverse effects compared to corticosteroids. To date, however, the underlying mechanism of natural ACTH on macrophage function remains unknown necessitating further explorations.

In the present study, we evaluated the efficacy of natural ACTH on acute gout in mice, then evaluated its regulatory function in THP-1 cells following stimulation by MSU. Results from animal experiments revealed that subcutaneous injection of a high concentration of natural ACTH effectively alleviated swelling and inflammation in mice joints caused by MSU crystal stimulation. Although a low concentration of natural ACTH could not significantly ameliorate the swelling, it still prevented accumulation of inflammatory cells. Additionally, we found no significant changes in the level of cortisol in mice blood after treatment, indicating that natural ACTH does not affect cortisol synthesis. Therefore, we explored the mechanism through which natural ACTH alleviates acute gout-induced inflammation through macrophages. Results from both in vivo and in vitro studies demonstrated that natural ACTH effectively alleviates inflammation in the joints of mice with acute gout and affects the polarization and phagocytosis of macrophages to some extent. Overall, these findings indicate that ACTH functions differently from typical corticosteroids like dexamethasone.

## 2. Materials and Methods

### 2.1. Patients and Treatment

Five gout patients who satisfied the preliminary criteria described by the American Rheumatism Association (ACR) for acute arthritis of primary gout and the 2015 ACR/European League Against Rheumatism (EULAR) gout classification were included in this study. This study was approved by the Ethics Committee of the Department of Huashan Hospital, Fudan University (No. 2021–495), and the patients provided written consent for their biological material to be used for research. Analysis of patient data as well as results from in vitro and in vivo experiments indicated that natural ACTH effectively alleviates inflammatory response by inhibiting the aggregation of inflammatory cells and changing the function of macrophages. At the transcriptional level, this effect is different from that exerted by dexamethasone.

### 2.2. Methods

#### 2.2.1. Establishment of a Mouse Model

Six-week-old C57BL/6 mice were bought from Shanghai JieSiJie Laboratory Animal Limited Corporation and maintained under sterile conditions with feed and water provided ad libitum. All experiments involving animals were conducted in accordance with the guidelines approved by the Animal Committee of Fudan University. A gout mouse model was established using MSU crystals. Briefly, mice were first divided into three groups, anesthetized via inhalation of 3% isoflurane (Forane; Abbot, Chicago, IL, USA), followed by intra-articular injection with 50 *μ*l (1 mg) of MSU suspension in normal saline in the right footpad. Control mice were injected with 50 *μ*l of normal saline into their left footpad. Thirty minutes later, 800 *μ*l of 0.25 U/ml and 2.5 U/ml of natural ACTH was subcutaneously injected into each mouse. Next, blood was collected from each group of mice after 8 hours before the mice were sacrificed. The blood was then centrifuged for 15 minutes at 3000 rpm under 4°C to collect serum. Prior to injection of MSU crystals, we measured the thickness of the hind joint (3 times) using a caliper, then calculated its average. This measurement was performed again after 8 hours and compared with the initial value. Joint swelling was denoted by the ratio of average right joint thickness relative to that of the left.

#### 2.2.2. Histochemical Analysis

Mice were sacrificed after joint index evaluation, and their joint tissues were collected. These were fixed, embedded in paraffin, and sectioned to 5-*μ*m thick slices followed by haematoxylin and eosin (H&E) staining.

#### 2.2.3. Enzyme-linked Immunosorbent Assay (ELISA)

The concentration of serum cortisol and factors, including IL-1*β*, IL-6, TNF-*α*, and TGF-*β* in cells, were quantified using an ELISA kit (eBioscience).

#### 2.2.4. Natural ACTH

Natural ACTH (25 U per ampoute) was purchased from Shanghai NO. 1 Biochemical and Pharmaceutical Limited Corporation and diluted into various concentrations using triple-distilled water.

#### 2.2.5. Cell Cultures and Treatment

Tohoku Hospital Pediatrics-1(THP-1) cells were bought from the National Collection of Authenticated Cell Cultures and cultured in RPMI 1640 culture medium supplemented with 10% FBS. The cultures were incubated under humid conditions with 5% CO_2_ and at 37°C and subcultured after every 48 to 72 hours. Upon sufficient growth, the cells were transferred to cell culture plates, then PMA was added at a ratio of 1 : 10000 followed by a 48-hour incubation to induce conversion to macrophages. The culture medium was changed prior to experiments and disposed of through different methods as previously described. Next, the cells were incubated with 100 *μ*g/ml of MSU crystals for stimulation and 30 minutes later, exposed to 1.25 × 10^−4^ and 2.5 × 10^−4^ U/ml natural ACTH and 100 nM dexamethasone, respectively. Cells were collected after 48 hours of incubation for subsequent experiments.

#### 2.2.6. Flow Cytometry

Single-cell suspensions were stained by anti-Arg-1 (17-3697-82; eBioscience) and anti-iNOS (12-5920-82; eBioscience) antibodies, at a ratio of 1 : 100, and incubated for 40 minutes at 4°C under darkness. Next, the contents were incubated with FITC-Latex Beads (500290; Cayman Chemical), followed by analysis on the Canton C6 flow cytometer. The resulting data were analyzed by FlowJo.

#### 2.2.7. Intracellular Reactive Oxygen Species (ROS) Determination

Levels of intracellular ROS were determined using the Reactive Oxygen Species Assay Kit (DCFH-DA, Beyotime, Jiangsu, China). Briefly, the culture medium was aspirated from the cells after stimulation, DCFH-DA was added to a serum-free medium at a ratio of 1 : 1000 followed by a 20-minute incubation at 37°C. The contents were washed 3 times with the serum-free medium, and the cells were subjected to fluorescence microscopy and flow cytometry.

#### 2.2.8. Determination of Mitochondrial Function

Variations in the opening of mitochondrial permeability transition pores (mPTPs) were detected by a Mitochondrial Permeability Transition Pore Assay Kit (Beyotime, Jiangsu, China), according to the manufacturer's instructions. Briefly, the culture medium was aspirated from the cells after stimulation followed by 1 or 2 washes with PBS. Appropriate amounts of Calcein AM were added to the cells, followed by 30-45-minute incubation at 37°C under darkness. Fresh medium was then added to the contents, followed by another 30-minute incubation at 37°C under darkness. Finally, the medium was aspirated and cells were washed 2-3 times with PBS followed by observation and detection via fluorescence microscopy and flow cytometry, respectively.

#### 2.2.9. Statistical Analysis

Statistical analyses of data from all experiments (in triplicate) were performed using GraphPad Prism 8 (GraphPad Software, La Jolla, CA, USA), and expressed as means ± standard deviation (SD). Repeated measures of analysis of variance (ANOVA), followed by a post hoc test, were used to compare means among groups. Data followed by *P* < 0.05 were considered statistically significant.

### 2.3. Quantitative Real-time Polymerase Chain Reaction (qRT-PCR)

Total RNA was first extracted from samples using the Trizol reagent, according to the manufacturer's instructions, then converted to complementary DNA (cDNA) using the ReverTraAce kit (Toyobo). QRT-PCR was conducted on the CFX96 Touch Real-Time PCR system (Bio-Rad) using a SYBR Green Kit (Roche). Relative mRNA expression of target genes in the samples was calculated using the 2^−△△^Ct method and normalized to that of mouse GAPDH as an internal amplification control. Primer sequences were as follows:

- 5′-CCAAATTGCTGCATGAACCAG-3′ (forward)
- 5′-TGCTTCCGAGGAGTGTCTTTC-3′ (reverse) (for XDH gene);
- 5′-TGCTGCCCTTTGACAACCTG-3′ (forward)
- 5′-TGCTCCCGAAGTAAGAGGGT-3′ (reverse) (for MPO gene);
- 5′-TTGTTTGGTTAGGGCTGAATGT-3′ (forward)
- 5′-GCCAATGTTGACCCAAGGATTTT-3′ (reverse) (for NOX1 gene);
- 5′-ACCGTGGAGGAGGCAATTAGA-3′ (forward)
- 5′-TGGTTGCATTAACAGCTATCCC-3′ (reverse) (for NOX3 gene);
- 5′-AGAAGATTCGGAAACAACAGCA-3′ (forward)
- 5′-GCTGGATCATTAGTTCTTGAGCC-3′ (reverse) (for NR1H2 gene);
- 5′-TTCTTTGCATTAGCCTCATCCTT-3′ (forward)
- 5′-CGTGCTGATTCCTTTTGGGC-3′ (reverse) (for IL-37 gene);
- 5′-GATCTTCGCTGCGATCAACAG-3′ (forward)
- 5′-CGTGCATTATCTGAACCCCAC-3′ (reverse) (for NLRP3 gene);
- 5′-GACTTTAAGGGTTACCTGGGTTG-3′ (forward)
- 5′-TCACATGCGCCTTGATGTCTG-3′ (reverse) (for IL-10 gene);
- 5′-CTCTGGCGTAGAGCTATCACT-3′ (forward)
- 5′-AGGCTGGGTTGGTGAAAACA-3′ (reverse) (for MerTK gene);
- 5′-CCTCCTGTCTAGTCGGTTTGG-3′ (forward)
- 5′-TCGAGCACCCTGTACCATTGA-3′ (reverse) (for Fc*γ*RIIIA gene);
- 5′-CATCTCCTTGCGATTCTGTTTTG-3′ (forward)
- 5′-CCATTCCGAGTGCTCCTGA-3′ (reverse) (for PTX3 gene);
- 5′-GACTGTCCTCGTGTGGTTTTG-3′ (forward)
- 5′-GGCTGCCCAGCATATCAGAT-3′ (reverse) (for MC2R gene);
- 5′-GCCAACACTGCCTAATGGCT-3′ (forward)
- 5′-AACCTCGGGCTTGATGAAGAC-3′ (reverse) (for MC3R gene);
- 5′-TCTGAGTCTGTATGGAGTGACAT-3′ (forward)
- 5′-CCAAGTCGTTCACATCTAGTTCA-3′ (reverse) (for PGC-1*α* gene);
- 5′-TGGACGCAGGTTCTCCAAAC-3′ (forward)
- 5′-CCGGCTCGCAGTAGGTAAC-3′ (reverse) (for SMAD3 gene);
- 5′-GGTAGCTGAGTTTGACTTCCG-3′ (forward)
- 5′-GACAGCATCCCTGTTGACCTT-3′ (reverse) (for GAS6 gene).

## 3. Results

Our preliminary results showed that natural ACTH not only effectively alleviated inflammation in mice joints but also weakened phagocytosis in macrophages, phenomena that may have been caused by polarization of M2 macrophages and promoted by natural ACTH. Unsurprisingly, natural ACTH inhibited the ability of MSU-stimulated THP-1 cells to secret M1 inflammatory factors, an effect that was similar to that observed in dexamethasone. Interestingly, the addition of natural ACTH induced upregulation of Arg-1 in THP-1 cells, suggesting that this drug can inhibit inflammation by promoting polarization of M2 macrophages.

### 3.1. Natural ACTH Rapidly Alleviates Inflammation Caused by Acute Gout in Patients, with No Effect on Cortisol and ACTH Levels

We evaluated the level of pain in the 5 recruited patients after treatment with natural ACTH via a VAS pain scale and found that on average, all of them experienced less pain to some extent for 6–12 hours. Their cortisol and ACTH levels in blood were within normal ranges 24 hours after treatment. Detailed results are shown in Table 1.

### 3.2. Natural ACTH Alleviates Swelling and Inflammation in Mice Joints with No Effect on Cortisol Levels

We established an acute gouty arthritis mouse model by injecting MSU crystals into their joints, followed by detection. We observed significantly higher swelling in the right joint of MSU-treated mice relative to those in the control group and the other joints of the treated mice. Subcutaneous injection of ACTH (0.25 U/ml per mouse) had no significant effect on joint swelling, while 2.5 U/ml per mouse effectively alleviated the phenomenon (Figure 1(a)). *H* and *E*-stained sections revealed severe inflammation in the joints of MSU-treated mice, which was higher than those treated with natural ACTH (Figure 1(b)). ELISA readings revealed no significant differences between the groups with regard to cortisol concentration in blood (Figure 1(c)).

### 3.3. Natural ACTH Suppresses Phagocytosis in Macrophages

We incubated THP-1 cells with different concentrations of natural ACTH, with dexamethasone as the control drug, and assessed changes in phagocytosis. Results indicated that both natural ACTH and dexamethasone significantly inhibited phagocytosis compared to treatment with MSU alone. Notably, a higher natural ACTH concentration resulted in a higher inhibition effect (Figure 2(a)). Moreover, both natural ACTH and dexamethasone effectively inhibited the ability of macrophages to engulf FITC-Latex Beads relative to the control group in a concentration-dependent manner (Figure 2(b)).

### 3.4. Natural ACTH Promotes Polarization of M2 Macrophages and Downregulates Expression of Proinflammatory Factors

MSU crystals stimulated THP-1 cells to release inflammatory factors like IL-1*β* (Figure 3(a)), IL-6 (Figure 3(b)), and TNF-*α* (Figure 3(c)), although treatment with natural ACTH and dexamethasone significantly downregulated expression of these factors. Interestingly, the levels of TGF-*β* did not change in the presence of natural ACTH and only decreased upon treatment with dexamethasone (Figure 3(d)). We used flow cytometry to detect and analyze polarization markers, such as iNOS/Arg-1, and found that MSU crystals stimulated THP-1 cells thereby causing significant polarization of M1 macrophages. A low natural ACTH concentration effectively inhibited the trend and promoted polarization of M1 to M2 macrophages, while a higher concentration resulted in no significant change (Figure 3€).

### 3.5. Natural ACTH Suppresses ROS Production in Gouty Macrophages and Protects Mitochondrial Function by Inhibiting XDH Production

MSU crystals significantly elevated ROS production, while both natural ACTH and dexamethasone reversed the phenomenon (Figure 4(a)). We further explored whether natural ACTH could protect the mitochondrion by detecting the opening of mPTP and found that exposure to MSU crystals promoted this process (Figure 4(b)). Interestingly, natural ACTH and dexamethasone effectively reversed this function. Besides, natural ACTH generated a stronger protective effect than dexamethasone, which was positively correlated with its concentration. Furthermore, qRT-PCR results revealed significant downregulation of XDH in the group treated with natural ACTH, while NOX3 was significantly downregulated in the dexamethasone group (Figure 4(c)).

### 3.6. Natural ACTH Regulates Transcription of Inflammatory-related Genes via a Different Anti-Inflammatory Mechanism to That of Dexamethasone

Results from PCR array analysis used to evaluate transcriptional differences between natural ACTH and dexamethasone during anti-inflammatory responses are shown in Figure 5(a). Particularly, we observed differences between natural ACTH and dexamethasone with regard to metabolism (Figure 5(b)), inflammation (Figure 5(c)), phagocytosis (Figure 5(d)), melanocortin receptors (Figure 5(e)), and other related genes (Figures 5(f)–5(j)). Notably, natural ACTH did not affect the expression of most genes, although it upregulated some such as NR3C1, NR1H2, IL-37, Fc*γ*RIIIA, and GAS6 and downregulated others like NLRP3, MC2R, and MC3R. On the other hand, dexamethasone significantly affected the expression of ANGPTL4, PDP1, PDHA1, VDR, IL1RN, IL-10, MERTK, PTX3, DDIT4, and SMAD3 relative to natural ACTH.

## 4. Discussion

Upon the development of acute gout in patients, macrophages within the articular cavity and those transformed from monocytes existing in blood engulf MSU, thereby secreting proinflammatory factors that induce inflammation [16]. Consequently, this phenomenon plays an important role in the development and progression of inflammation. To ascertain this concept, we treated THP-1 cells with natural ACTH and dexamethasone that had been stimulated by MSU and found that both drugs significantly inhibited the phagocytic function of these cells. Notably, this effect occurred in a concentration-dependent manner. In order to verify that the observed inhibitory function on THP-1 cells was not specifically due to MSU, we used FITC-Latex Beads to detect the phagocytic ability of THP-1 cells via fluorescence microscopy and flow cytometry and found that Latex Beads with FITC could be engulfed by macrophages. These results corroborated those from MSU stimulation, affirming that natural ACTH effectively inhibits phagocytosis of THP-1 cells and further suppressed MSU-stimulated secretion of inflammatory factors.

Apart from phagocytosis, macrophages have been shown to develop into proinflammatory M1 type during the early period of inflammation [17]. Previous studies have demonstrated that MSU crystals can stimulate the cells to secrete IL-1*β*, IL-6, and TNF-*α* to induce inflammatory infiltration and drive persistence of gouty inflammation [18]. The function of immune cells largely depends on their metabolic activity. Therefore, the cells need to develop metabolic adaptation in order to support their various immunological functions. Macrophages, which play a crucial role in innate immunity, are strictly regulated by the metabolic pathway and corresponding metabolites [19]. In fact, the role of mitochondrion regulating immune cell function cannot be ignored and is considered the center for cell metabolism. Numerous regulatory mechanisms have been gradually revealed over the years. For example, studies have shown that mitochondrial reactive oxygen species (mtROS), which are generated during the process of electron transfer chain, may trigger innate immune signals and damage the cells, the extent of which depends on the volume of mtROS and the time of occurrence [20]. Additional evidence has demonstrated that inflammation may eleviate ROS production in macrophage mitochondria, thereby inhibiting oxidative phosphorylation function, which is indicative of impaired mitochondrial function [21, 22].

In the present study, we hypothesized that natural ACTH could protect the mitochondria of THP-1 cells to some extent, thus performed experiments to verify this. Results revealed high ROS production in the mitochondria of THP-1 cells upon MSU stimulation, although this process was significantly inhibited after treatment with natural ACTH and dexamethasone. mPTP, a group of protein complex that exists between the inner and outer mitochondrial membranes, is a type of nonspecific channel that plays a significant role in cell survival and apoptosis and is also involved in various fields, such as ischemia/reperfusion, cancer, aging, and neural degeneration [23]. Notably, mPTP allows ions with a relatively low molecular mass to freely permeate under physiological conditions; thus, it maintains the mitochondrial membrane potential and the balance of ions both within and outside the cells by driving ATP synthase through oxidative phosphorylation. However, apoptotic signals promote full opening of mPTP, which makes soluble matter to permeate nonselectively, thereby generating an ion imbalance and membrane potential depolarization and causing apoptosis or necrosis [24, 25]. Since mPTPs can be targeted to detect impairment of mitochondrial function, we measured the protective function of natural ATCH on mPTPs. Results revealed that numerous mPTPs existing in THP-1 cells opened upon MSU-mediated stimulation, indicative of damage to the mitochondrial function. In contrast, both natural ACTH and dexamethasone reversed this phenomenon, although ACTH had a superior effect suggesting that it offers better protection to the mitochondria in THP-1 cells and maintains the functionality of mPTPs relative to dexamethasone. As qRT-PCR-based analysis of gene expression in XDH, MPO, NOX1, and NOX3, all of which regulate ROS production, revealed that natural ACTH downregulated XDH expression in MSU-stimulated THP-1 cells. This gene has previously been implicated in conversion of products of purine metabolism into uric acid [26]. Overall, these results indicated that natural ACTH inhibits production of uric acid and protects mitochondrial function. However, further studies are needed to prove this aspect.

Although glucocorticoids are effective in treating patients with gout, various corresponding side effects, such as central obesity, infection, calcium loss, osteoporosis, diabetes, and stomach ulcers, cannot be ignored [27]. In fact, avoiding these adverse events during treatment remains a huge concern. We hypothesize that there may be some differences between ACTH and glucocorticoids with regard to the effect of treatment. Moreover, whether natural ACTH is a better choice for the treatment of acute gout remains unclear. Based on PCR array results, we selected and analyzed the expression of genes regulating metabolism, inflammation, and phagocytosis among others associated with anti-inflammatory effects. Results showed that natural ACTH did not significantly affect the expression of metabolism-related genes, except NR3C1, a receptor of glucocorticoids within cells. We speculated that this gene may have a permissive effect on glucocorticoids. Dexamethasone upregulated the ANGPTL4 expression but downregulated those of PDP1, PDHA1, NR3C1, and VDR, suggesting that it may have a negative effect on metabolism of sugars, lipids, proteins, and osteocytes but plays an anti-inflammatory role [28, 29]. With regard to inflammatory-related genes, natural ACTH did not significantly affect expression of IL1RN and IL10. However, its treatment upregulated NR1H2 and IL37 but downregulated that of NLRP3. In addition, dexamethasone upregulated expression of IL1RN and IL10 but had no significant effect on expression of the others. This might suggest that ACTH and dexamethasone employ different anti-inflammatory mechanisms during the regulation of the hepatic acute phase and immune responses [25, 26]. Furthermore, natural ACTH did not significantly affect the expression of phagocytosis-related genes, but dexamethasone upregulated all of them. These phenomena may be attributed to the function of engulfing apoptotic cells like MERTK [27], innate resistance to pathogens, and inflammatory reactions such as PTX3 [28] and FccRIIIA [29]. Next, we analyzed the expression of some genes regulating hormones and their receptor pathways, such as classic receptors of ACTH on macrophages MC2R and MC3R, a kind of proto-oncogene BCL6 [35], DNA damage-induced transcription protein DDIT4 [36], a transcriptional coactivator for steroid receptors and nuclear receptors PGC-1*α* [37], an intracellular signal transducer and transcriptional modulator SMAD3 [38], and a ligand for tyrosine-protein kinase receptors GAS6 [39]. Results showed that natural ACTH exerted similar therapeutic effects as dexamethasone, although both did not significantly affect the expression of most of these genes.

## 5. Conclusion

To sum up, our results indicated that natural ACTH alleviates inflammatory responses and regulates macrophages in acute gout. There are still some shortcomings in this experiment, such as the number of clinical samples and the evaluation criteria for patients can still be improved. Notably, natural ACTH regulates gene transcription in a different fashion to corticosteroids. Taken together, these results indicate that natural ACTH is an effective therapeutic option for patients who may encounter problems with NSAIDs, steroids, or colchicine. Further studies are needed to determine the differences in efficacies between natural ACTH and corticosteroids, to ascertain whether natural ACTH is a safe alternative to corticosteroids.

## Figures and Tables

**Figure 1:** Natural ACTH alleviates swelling and inflammation in mice joints. (a): swelling of mice joints denoted by the ratio of average thickness in the right joint relative to the left joint. (b): histological changes of the right joint of mice with acute gouty arthritis. Bars = 2.5 mm (left) and 250 *μ*m (right). (c): ELISA results indicating the level of cortisol in mice serum (pg/ml). *n* = 3; ^*∗*^*P* < 0.05; ^*∗∗*^*P* < 0.01; ^*∗∗∗*^*P* < 0.001; n.s., no significance. ELISA: enzyme-linked immunosorbent assay.

**Figure 2:** Natural ACTH inhibits phagocytosis of THP-1 cells. (a) Flow cytometry results, after 48 hours, showing macrophages with different degrees of phagocytic inhibition after treatment with natural ACTH and dexamethasone. (b) The ability of macrophages to phagocytose Latex Beads was suppressed by natural ACTH and dexamethasone treatment. Data presented are means ± SEM for at least three independent experiments. ^*∗*^*P* < 0.05; ^*∗∗*^*P* < 0.01; ^*∗∗∗*^*P* < 0.001; ^*∗∗∗∗*^*P* < 0.0001; n.s., no significance. ACTH: adrenocorticotropic hormone.

**Figure 3:** Natural ACTH converts M1 to M2 macrophages. (a) ELISA results showing concentration of IL-1*β*, IL-6, TNF-*α*, and TGF-*β*. (b) Profiles of polarization determined by the ratio of iNOS fluorescence intensity to that of Arg-1. Data presented are means ± SEM for three independent experiments. ^*∗*^*P* < 0.05; ^*∗∗*^*P* < 0.01; ^*∗∗∗*^*P* < 0.001; n.s., no significance. ELISA: enzyme linked immunosorbent assay; IL-1*β*: interleukin-1*β*; IL-6: interleukin-6; TNF-*α*: tumor necrosis factor-*α*; TGF-*β*: transforming growth factor-*β*; iNOS: nitric oxide synthase; Arg-1: arginase-1.

**Figure 4:** Natural ACTH downregulates ROS production in macrophages and inhibits the opening of mPTP. (a) Fluorescence microscopy images showing intensity of ROS production as shown by MFI. (b) Fluorescence microscopy and flow cytometry results showing that intensity was negatively correlated with damaged mitochondrial function. Bars = 100 *μ*m. (c–f): qRT-PCR results showing expression of related genes. ^*∗*^*P* < 0.05; ^*∗∗*^*P* < 0.01; n.s., no significance. ROS: reactive oxygen species; MFI: Median Fluorescence Intensity; qRT-PCR: quantitative Real-time PCR.

**Figure 5:** Natural ACTH regulates transcription of inflammatory-related genes via a different mechanism to that of employed by dexamethasone. (a) A heat map showing differences in the effect of natural ACTH and dexamethasone on gene transcription of THP-1 cells. (b–j): Expression profiles for some of the related genes. ^*∗*^*P* < 0.05; ^*∗∗*^*P* < 0.01; ^*∗∗∗*^*P* < 0.001; n.s., no significance. ACTH: adrenocorticotropic hormone. THP-1: Tohoku Hospital Pediatrics-1.

**Table 1:** Natural ACTH can quickly alleviate inflammation without affecting the level of cortisol and ACTH.

Patient	Sex	Age	VAS rating									Blood cortisol level (normal range) ^*∗∗*^, ug/dL	Blood ACTH level (normal range) ^*∗∗*^, ug/dL
			0 hours	6 hours	12 hours	24 hours	48 hours	72 hours	4 days	5 days	6 days		
1	Male	33	6	5	3	2	2	2	4 ^*∗*^	2	1	4.88 (2.3 ∼ 11.9)	19.45 (3 ∼ 32)
2	Male	30	3	3	2	2	2	1	1	0	0	7.13 (2.3 ∼ 11.9)	8.47 (3 ∼ 32)
3	Male	27	10	8	5	7	5	5	5	3	3	5.54 (2.3 ∼ 11.9)	15.17 (3 ∼ 32)
4	Male	54	8	6	8	6	6	5	4	3	2	18.31 (6.2 ∼ 19.4)	19 (6 ∼ 48)
5	Male	40	7	6	6	4.5	4	4	4.5	4	2.5	12.45 (6.2 ∼ 19.4)	23.6 (6 ∼ 48)

The pain VAS (0H-6 d) of five acute gout patients who were treated with natural ACTH and the level of cortisol and ACTH in their blood. For pain intensity, the scale is anchored by “no pain” (a score of 0) and “worst imaginable pain” (a score of 10). Patients can choose one score between 0 and 10 to describe the pain they are suffering. A score of 1 to 3 represents that there is a slight pain and the patients can bear it; a score of 4–6 indicates that the pain can also be tolerated although it may affect the quality of sleep; and a score of 7–10 means patients cannot tolerate the gradually strong sense of pain. ^∗^: patients once carried heavy objects during this period. ^∗∗^: blood tests were performed 24 hours after the treatment of natural ACTH. Variations displayed in the level of cortisol and ACTH were due to the circadian rhythm, and the results may differ slightly when detected in different periods.

## Data Availability

The datasets used and/or analyzed during the current study are available from the corresponding author on reasonable request.

## Abbreviations

ACTH: Adrenocorticotropic hormone
ANGPTL4: Angiopoietin-related protein 4
Arg-1: Arginase-1
ATP: Adenosine-triphosphate
AXL: Anexelekto
BCL6: B-cell lymphoma 6
CRF: Corticotropin-releasing factors
DCFH-DA: 2, 7-dichlorodi-hydrofluorescein diacetate
DDIT4: DNA damage inducible transcript 4
ELISA: Enzyme-linked immunosorbent assay
Fc*γ*RIIIA: Low-affinity immunoglobulin gamma Fc region receptor III-A
FITC: Fluorescein isothiocyanate
GAS6: Growth arrest-specific protein 6
HE: Hematoxylin-eosin staining
IL-1*β*: Interleukin-1 *β*
IL1RN: Interleukin 1 receptor antagonist
IL-6: Interleukin-6
IL-10: Interleukin-10
IL-37: Interleukin-37
iNOS: Nitric oxide synthase inducible
MC-2R: Melanocortin 2 receptor
MC-3R: Melanocortin 3 receptor
MERTK: MER proto-oncogene tyrosine kinase
MPO: Myeloperoxidase
mPTP: Mitochondrial permeability transition pore
mTOR: Mammalian target of rapamycin
MSU: Monosodium urate
NLRP3: NLR family pyrin domain containing 3
NOX1: NADPH oxidase 1
NOX3: NADPH oxidase 1
NR1H2: Nuclear receptor subfamily 1 group H member 2
NR3C1: Nuclear receptor subfamily 3 group C member 1, glucocorticoid receptor
NSAIDs: Nonsteroidal anti-inflammatory drugs
PBS: Phosphate buffered saline
PDHA1: Pyruvate dehydrogenase E1 subunit alpha 1
PDP1: Pyruvate dehydrogenase phosphatase 1
PGC-1*α*: Peroxisome proliferator-activated receptor gamma coactivator 1-alpha
PMA: Phorbol-12-myristate-13-acetate
PTX3: Pentraxin-related protein PTX3
qRT-PCR: Quantitative real-time PCR
ROS: Reactive oxygen species
RPMI: Roswell Park Memorial Institute
SMAD3: Others against decapentaplegic homolog 3
TGF-*β*: Transforming growth factor-*β*
THP-1: Tohoku Hospital Pediatrics-1
TNF-*α*: Tumor necrosis factor-*α*
TYRO3: Tyrosine-protein kinase 3
VAS: Visual analogue scale
VDR: Vitamin D3 receptor
XDH: Xanthine dehydrogenase/oxidase.
